RETRACTED

# Force Platform-Based Intervention Program for Individuals Suffering with Neurodegenerative Diseases like Parkinson

**DOI:** 10.1155/2022/1636263

**Published:** 2022-01-17

**Authors:** Javed Ahmed Ujjan, William Morani, Naz Memon, Sugumar Mohanasundaram, Shibili Nuhmani, Bhupesh Kumar Singh

**Affiliations:** ^1^College of Animal Sciences & Technology, Northwest A & F University, China; ^2^Department of Zoology, Shah Abdul Latif University, Khairpur, Sindh, Pakistan; ^3^University of Heidelberg, Germany; ^4^Mehran University of Engineering and Technology, Jamshoro, Pakistan; ^5^Department of Biochemistry, Sri Sankara Arts and Science College, Enathur, Kanchipuram, Tamilnadu, India; ^6^Department of Physical Therapy, Imam Abdulrahman Bin Faisal University, Dammam, Saudi Arabia; ^7^Arba Minch Institute of Technology, Arba Minch University, Ethiopia

## Abstract

The term “neurodegenerative disease” refers to a set of illnesses that primarily affect brain's neurons. Substantia nigra (a midbrain dopaminergic nucleus) with lack of hormone called dopamine causes Parkinson's disease (PD), a neurological disorder. PD leads to tremor, stiffness, impaired posture and balance, and loss of automatic movements. Patient with Parkinson's often develops a parkinsonian gait that includes a tendency to lean forward, small quick steps as if hurrying forward, and reduced swinging of the arms. They also may have trouble initiating or continuing movement. Gait analysis is often used to diagnose neurodegenerative illnesses and determine their stage. In this study, we attempt to investigate postural balance, and of gait signals for Parkinson's patients, also, we incorporate interim rehabilitation technique. We included 25 PD patients who had 2.5 to 3 IV score of Hoehn and Yahr scale. A ten-minute walk test has been performed to observe primary and secondary results of dual task interference on gait velocities, and gait time motion vector for right and left legs was observed. Two experimental ground conditions include three conditions of trunk alignment, that is, erect on a regular basis (RE), trunk dorsiflexion 30° (TF1), and trunk dorsiflexion 50° (TF2) were analysed. We identified the walking speed of PD patients was decreased, and trunk dorsiflexion variables influence the gait pattern of Parkinson's disease patients, where higher 95% CI for TF1 condition was reported. The regular erect trunk showed swing time reduction (0.7%) in PD, so the higher unified PD rating scale (UPDRS) values have significant difference in swing phase time in Parkinson's patients. The average Hoehn and Yahr scale (H&Y scale) was 4.3 ± 2.5 reported in the study participants. In a 10-week follow-up evaluation, the stance duration was shown to be substantial, as was the slower speed gait in the baseline condition. Excessive flexion was discovered in our investigation at the lower limb joints, particularly the knee and ankle. Patients with Parkinson's disease had similar maximum dorsiflexion and minimum plantarflexion values in stance. The trunk fraction conditions were found significant in patients after rehabilitation training. The best response to rehabilitation treatment was seen when the trunk was rotated. When steps and posture distribution analysis performed, we found that the trunk flexure 1 (*p* < 0.05), and trunk flexure 2 (*p* < 0.01) were shown significant values. When GRF threshold characteristics are employed, mean accuracy improves by 52%. Regardless of gait posture, the step regular trunk flexure had significantly higher posture than the corresponding level steps, with a considerable rise in the 50 in trunk dorsiflexion 2 gait relative to the step “L.” This study shows that there was some significant improvement observed in the gait parameters among patients with PD's which shows positive impact of the intervention. Furthermore, rehabilitation programmes can aid and improve poor gait features in patients with Parkinson's disease, especially those who are in the early stages of the condition. This gait and balance research provides a rationale for intervention treatments, and their use in clinical practise enhances evidence of therapeutic efficacy. However, prolonged follow-up is needed to determine whether the advantages will remain all across disease's course, and future studies may recommend a specific rehabilitation technique based on gait analysis results.

RETRACTED

## 1. Introduction

Neurodegenerative diseases (NDs) fall into one of those kinds of diseases where cure does not prevail. One suffering from these diseases faces decline in health and partial or complete whose decline can partially or complete set back with normal course of life. Loss of neurons and axons is considered as major reason for onset as well as progression of such disease. The loss of axons and the development of abnormalities along with the decreasing neurons in the central nervous system are main causes of NDs [1]. Ageing, neuronal inflammation, and free radical toxicity (i.e., oxidative stress) are all thought to be linked to NDs, which can lead to cognitive decline and motor dysfunction [2]. A few examples of NDs such as spinal muscular atrophy, Alzheimer's disease, Huntington's disease, and amyotrophic lateral sclerosis are to name a few [3]. PD is considered as the 2nd most commonly prevailing neurodegenerative disease, which comprises two forms, one is familial, and the other is idiopathic forms.

RETRACTED

This illness is identified as the decreasing of dopaminergic and noradrenergic neurons of the ventral midbrain and locus coeruleus, respectively, regardless of the aetiology; however, by the time symptoms appear, a significant number of neurons in both locations have been destroyed. Neuroprotective medicines and treatments are thought to be best combined with far more sensitive and precise biomarker tests that can predict and detect individuals at risk or early-stage risk screening of individuals which can be started later as disease-altering therapy at the earliest [4]. Parkinson's disease is mainly identified by reduced dopamine production [5, 6], which leads to alterations in the cortical area, which is involved in movement planning and sequencing [7].

The diagnosis or expression of PD is monitored, which clinical evaluation-based test takes into account numerous subjective factors. The lack of quantifiable biomarkers for diagnosis and symptom monitoring results in considerable out-of-pocket health costs, both direct and indirect. The state of the art of diagnostic criteria [8, 9]exist nearly 20% error rate [10]. Gait deficits are the most visible and prevalent symptom of Parkinson's disease, and they are recognised to be predictive of future motor, psychosocial, and cognitive impairment. However, identifying important biomarkers and, as a result, materialising rehabilitation strategies and tactics necessitate a detailed understanding of muscular activity which causes gait impairment as well as the therapeutic interventions impact on motor behaviour [11–13]. As the illness develops, numerous gait abnormalities emerge, displaying distinct patterns of gait disruptions [14], reduced speed, shorter step length [15], and shuffling steps, requiring stronger double limb support, more pace, discreetness in turns (i.e., turning blocks), and difficulties along with freezed gait [16], inferior balance, and postural controls. It is commonly noticed that with due course of time, many gait features get worse in PD.

Depending on type of NDs, it can result to be serious or life-threatening as most of them lack its prevention and cure. Early and timely onset of medication as well as treatment may not stop occurrence of advance PD but it may definitely provide support to patients by reliving pains, thus supporting one's mobility. Thus, here, in this study, we aim to collect gait signals for Parkinson's patients by Kistler quartz (piezo-electrical) force platform, with Bioware Software. For the percentile of force exertion, velocity, and auxiliary signal data collection, descriptive statistics were produced. ANOVA has been used for one-way (steps and postures) repeated where time blocks as a variant used to evaluate the effect of postures on force exertion metrics.

RETRACTED

Other objective analysis techniques include nonwearable sensors (NWS) like image processing (IP) and whole body scanner (3D motion) with markers on the particular location of body. The other types of optic sensors such as laser range scanners (LRS), infrared sensors, and time-of-flight (ToF) and stereoscopic vision cameras are also used. The semisubjective analysis techniques contain Timed 25-Foot Walk (T25-FW), Multiple Sclerosis Walking Scale (MSWS-12), Gait Abnormality Rating Scale (GARS), and Tinetti Performance-Oriented Mobility Assessment (POMA) tests [17].

The practical utility of the present research work is to compare the spatiotemporal and kinematic parameters of gait in PD patients. Semiquantitative rating scale methods provide a clinician-based quantification of disease risk; these scales do not provide objective quantitative measures. Therefore, no need to apply quantitative measures to evaluate motor function in parkinsonism. Gait analysis is one of the most commonly used instruments to examine locomotion. Gait analysis is a noninvasive, three-dimensional computerised, and widely used technique. Such type of advance techniques allows an objective evaluation of different gait parameters and provides accurate and reliable information of gait variation of PD patients. This reduces the error margin caused by subjective techniques [18].

In the present study, we have applied Hoehn and Yahr scale and unified PD rating scale for the disease severity evaluation. For group of 25 PD patients, gait velocity and time for left and right were measured by a 10-minute walk test along with three trunk alignment conditions.

## 2. Methodology

*Ethical clearance*. The Institutional Committee as well as a partnered hospital approved the data collection format and experimental techniques to prospectively gather detailed information on acute stroke patients in order to conduct this study. A signed informed consent form was required from each patient. The complete data collection procedure was carried out in accordance with the approved methodology and standards.

This is a cross-sectional study where an intervention was performed, and its assessment was done by collection of gait signal. For this study, clinical as well as an instrumental assessment for gait analysis was performed by collecting data at the day of enrolment for rehabilitation, and second set of data collection was done after 21 days of rehabilitation treatment.

### 2.1. Selection of Participants

#### 2.1.1. Sample

After screening from the exclusion and inclusion criteria, here, we recruit twenty-five patients for this study (Figure 1). The recruited participants were rehabilitated in the treatment centre of our collaborated university hospital.

RETRACTED

#### 2.1.2. Inclusion Criteria

Inclusion criteria are as follow: (1) those who are willing to participate, (2) those who went through neurological evaluation, (3) those who were about to start their rehabilitation treatment, (4) those whose medication was kept unchanged throughout the intervention, (5) idiopathic PD: (i) stage 2.5 or 3 scores IV on scale of Hoehn and Yahr [19] and (ii) presence of moderate FoG (unified PD rating III with Fog subscore of 2 or more), and (6) individuals who were able to meet the United Kingdom Brain Bank criteria for PD [20]. The examples for the United Kingdom Brain Bank criteria for PD includes Bradykinesia, muscular rigidity, 4-6 Hz rest tremor, and postural instability not caused by primary visual, vestibular, cerebellar, or proprioceptive dysfunction.

#### 2.1.3. Criteria for Exclusion

The following exclusion criteria were as follows:

1. Those who are not willing to participate: nonacceptability of a consent
2. Those who are not neurologically evaluated: patients identified and confirmed based on diagnostic tests and procedures by certified physician
3. Severe dyskinesias: such patients have abnormal, uncontrollable, and involuntary movements
4. Those whose PD medication about to change
5. Sensory dysfunction in limbs: the risk of falls and unbalancing are higher among this group, and temporal or spatial aspects of gait are not effectively measured by straight-line gait speed and number of steps
6. Orthopaedic problems affecting the limbs
7. Paroxysmal vertigo: most common cause of vertigo and leads to sudden sensation that you are spinning or that the inside of your head is spinning
8. Other severe medical problems or disease condition

Figure 1 shows the patient recruitment process.

### 2.2. Data Acquisition

#### 2.2.1. Primary and Secondary Outcomes

- The percentage (percent) of dual-task interference on gait velocity was the primary outcome measure for the 10-Meter Walk Test
- The standardized Berg Balance Scale (BBS) was used objectively determine a patient's ability (or inability) to safely balance during a series of predetermined tasks and scale consisting of a five-point ordinal scale ranging from 0 to 4, with 0 indicating the lowest level of function and 4 the highest level of function and takes approximately 20 minutes to complete (14 item) [21]
- Korean version-based Falls Efficacy Scale-International (KFES) was applied to patient's falls, which contains 16 items of gait, activities of daily living, and social activities. Each item was graded from 1 (not at all concerned) to 4 (very concerned which means having cognitive disquiet about the possibility of falling). Total scores were summated, with higher score indicating higher anxiety for falls [22]
- Berg Balance Scale (BBS) as well as Korean version-based Falls Efficacy Scale-International (KFES) were employed to assess the signal and dual task condition of gait speed. Describe the eight variables that are used to classify gait data from patient with Parkinson disorders. It displays the average of all characteristics' maximum and minimum values of the right and left gait obtained wherein the left feet had higher force

RETRACTED

### 2.3. Test Setup

For this study, few muscle position was identified such as tibialis anterior, upper trapezium, knee, lateral and anterior part of patella, midline spine, and soleus for monitoring the locomotion as upright position. Ag/AgCl pregelled electrodes were placed on this muscle for EMG signal. Ag/AgCl electrodes are classified as nonpolarizable electrodes (nonpolarizable electrodes to facilitate the electrochemical reactions and to reduce electrode-skin interface impedance) and considered as the universal electrodes in clinical measurements (e.g., ECG, EMG, and EEG) [23]. They are associated with low electrode-skin impedance, low noise, and low motion artifact [24]. For data normalisation, reference electrodes were inserted on both the arms and the spine (back), as well as an upright bare foot reading.

From force platform measurement as well as CoP displacement parameters, a Kistler, model number 9268AA, and an AD data log from BTS bio-engineering were utilised.

Kistler quartz (piezo-electrical) force platform: it is an advance classic piezoelectric measurement element for the measurement of force along a single axis. They can be used to measure compression or tensile force *F*_*z*_ or a shear force *F*_*x*,*y*_. It is used in various application such as in mounting technology, during the measurement of impact resistance, cutting forces and forming forces or in force plates, Weigh In Motion systems, and in crash-test setups.

The ground response forces which portrait the stabilometric vectors were measured using a piezoelectric-based platform. The piezoelectric platforms have been connected to amplifier control units of Kistler and a data collector. The platform acquired signals repeatedly for three times for 1 minute duration with 100 Hz frequency. Gait analysis was carried out on Kistler quartz (piezo-electrical) force platform, with Bioware Software 2812A (Kistler) used to analyse data Kistler (Kistler). An A–D data logger has been used to track the ground reaction forces that also show the stabilometric dimensions (BTS Bioengineering). Acquisitions of platform signals were done three times for a total of 60 seconds at frequency of 100 Hz. The weighted force distribution of standing position has been calculated using the root mean square (RMS) of three mutually perpendicular forces in *x*, *y*, *z*, directions. Force distribution was inbuilt gathered by RMS of *F*_*x*_, *F*_*y*_, and *F*_*z*_ forces in 3 directions, which has been based on the force platform signal procurement at feet. During a walking cycle, a unique pattern of force distribution was found.

RETRACTED

#### 2.3.1. Intervention

European physiotherapy guidelines for PD rehabilitation program was practiced by patients enrolled for the program [25]. This activity involved balance exercises, gait and physical exercise involved for prevention of inactivity, and reduction of pain or physical limitation, on an average-focussed patients involved in self-management aspects. Arm swings, foam walking, rolling over, large step walking, obstacle walking, climbing, bidirectional walking, taking turns in small, narrow, wide, and open space, standing, sitting, and walking on foam with and without agitations (pushes and pulls) to the chest, and lastly, sitting down were all part of this [26].

### 2.4. Design of Experiment and Parameter

The studied patient was allowed in standing or walking on the force platform, and initially, they obtained upright posture. The motion capture technique of force visual coding was recorded every movement [27]. The illuminators and sensors evaluate kinetics like displacement, velocity and acceleration, and angles. The ground reaction forces were processed by software, A/D board, and cabling. Subjects were given a 5-minute break between trials to reestablish steady circumstances. The trunk angle was measured in reference to the lab coordinate system's vertical axis by making connection of the L 5 marker (i.e., the midsection of L 5 and S1 junction) along with the C7 marker of the seventh cervical spinous process [28, 29]. Two experimental ground conditions include three condition trunk alignment that is erect on a regular basis (RE), trunk dorsiflexion 30° (TF1), and trunk dorsiflexion 50° (TF2). Both clinical and instrumental evaluations were used to assess gait at baseline (T0) and after having treatment of 10 weeks and rehabilitation (T1). Other studies that revealed outcome alterations found that the duration of treatment was consistent with the length of rehabilitation treatment.

Each week, the rehabilitation programme comprised three 60-minute sessions. According to predefined progression criteria, participants were encouraged to move through the programme by performing various exercises such as RoM exercise, stretching and strengthening of upper and lower limb, and improving balance of sitting, standing, and walking. Patient's neurological and functional characteristics were assessed using clinical measurements. The unified PD rating scale of II, III and Hoehn & Yahr phase system were used to assess the severity of the condition (Table 1).

RETRACTED

#### 2.4.1. Recordings from Instruments

*(1) Investigational Method*. Patients were asked to walk bare feet along a 12-meter corridor at a comfortable, self-selected pace while staring forward. Controls were asked to walk at their chosen tempo as well as at a slower pace. Because study's focus was on natural movement, broad qualitative guidelines were offered. All participants were trained for a few minutes before the recording session to acquaint themselves with the technique. For each patient, at least six trials were recorded for each trial. Each trial was separated by a 1-minute rest time to avoid muscular exhaustion.

*(2) Analysis*. The IBM SPSS 20.0 software has been used to conduct statistical analysis. For the percentile of force exertion, velocity, and auxiliary signal data collection, descriptive statistics were produced. One-way ANOVA used to determine the differences exists among the means obtained from different trials of steps and posture's gait also, for assessment of trends across categories. ANNOVA has been used for a one-way (steps and postures) repeated with time blocks as a variant to evaluate the effect of postures on force exertion metrics. The *p* value below 0.05 has been taken under consideration.

## 3. Results

Feature selection is a process of identifying and removing irrelevant and redundant features from datasets. Hundreds of thousands of features may be present in current databases. Some of them may be completely irrelevant, while others may contain redundant data. This can lead to extra issues as well as a longer classification processing time. This is especially useful for dealing with multidimensional data, allowing data mining algorithms to operate more efficiently and effectively. This problem can be addressed using a variety of approaches. More information can be found in [26].  Figure 2 shows the gait cycle of normal human.

The description for the recruitment of patients was bicentric observational study with a blind assessor. Gait analysis was performed as follows.

### 3.1. Measurements on the Force Platform

Gait analysis was carried out on Kistler quartz (Piezo-electrical) force platform, with Bioware Software (4.0.x Type 2812 A, Kistler) used to analyse data Kistler (Kistler). The ground reaction forces (GRF; *F*_*x*_, *F*_*y*_, *F*_*z*_), which indicate the dimension of stability, were monitored with an A–D data logger (BTS Bioengineering). At a sample frequency of 100 Hz, the acquisitions of platform signals were performed three times for a total of 60 seconds. The RMS of mutual perpendicular forces at *F*_*x*_, *F*_*y*_, and *F*_*z*_ coordinates has been used to determine the distribution of weighted force (in kgf) in standing posture. The flow chart depicting the patient recruiting processes is shown in Figure 3.

RETRACTED

### 3.2. Statistical Analysis

The SPSS 20.0 program package has been used to conduct the numerical investigation. For the percentile of force exertion, velocity, and auxiliary signal data acquisition, descriptive statistics were produced. The influence of postures on force exertion parameters was investigated using a one-way (steps and postures) repeated measure ANOVA with time blocks as a variant.

### 3.3. Design of Experiment and Parameter

The studied patient was allowed in standing or walking on the force platform, and initially, they obtained up right posture. The motion capture technique of force visual coding was recorded every movement. The illuminators and sensors evaluate kinetics like displacement, velocity and acceleration, and angles. The ground reaction forces were processed by software, A/D board, and cabling (Figure 4). Subjects were given a 5-minute break between trials to reestablish steady circumstances. By linking the L 5 marker and C7 marker to the lab coordinate system's vertical axis, the trunk angle was calculated (seventh cervical spinous process) [30, 31]. Two experimental ground conditions include three conditions trunk alignment that is erect on a regular basis (RE), trunk dorsiflexion 30° (TF1) and trunk dorsiflexion 50° (TF2). Both clinical and instrumental evaluations were used to assess gait at baseline (T0) and after treatment of 10 weeks followed by rehabilitation (T1). Other studies that revealed outcome alterations found that the duration of treatment was consistent with the length of rehabilitation treatment.

Clinical measures were used to assess patient's neurological and functional features. The severity of the illness was determined using the unified PD rating scale -II, III and Hoehn and Yahr phase system (Table 2).

*Program of Rehabilitation*. The European physiotherapy guidelines for PD (also known as The European Physiotherapy Guideline for PD, 2018) were followed by all of the patients who underwent physiotherapy treatment [29]. The programme emphasised self-management, preventing inactivity, and coping with fear of falling, as well as maintaining or improving global motor activities, transfer capabilities, balancing and manual activities, gait and pain management as well as control along with delaying the beginning of bodily restrictions.

1. Standing as well as moving on polystyrene foam with or and without trunk agitations (pushes and pulls)
2. Large-step walking and large-amplitude arm swings are some of the activities included in the study. During a normal gait cycle, approximately 60% and 40% of the time is spent in stance and swing, respectively

The span of these intermissions varies depending on your walking speed. Some small variations amongst the people in the study.

RETRACTED

Table 3 describes the eight variables that are used to classify gait data from patient with Parkinson disorders. It displays the average of all characteristics' maximum and minimum values of the right and left gait obtained wherein the left feet had higher force. The walking speed range between 0.6 and 1.75 (m/sec) recorded.

The arbiters of Parkinson's disease gait characteristics are listed in Table 4. The regression analysis shows that mean age, UPDRS rating scale, and trunk flexion variables influence the gait pattern of Parkinson's disease patients. Higher 95% CI value observed when trunk dorsiflexion at ~30° (3.8-6.7) followed by ~50° trunk dorsiflexion. Considerable knee flexion increases were seen across gait postures, as well as significant trunk dorsiflexion increases during regular erect trunk walking. The regular erect trunk showed swing time reduction (0.7%) in PD so, the higher UPDRS values have significant difference in swing phase time in PD patients. The Hoehn and Yahr scale (H&Y scale) has been used to determine how PD symptoms and impairment progressed [19]. The mean H&Y scale was 4.3 ± 2.5 reported in the study participants. The UPDRS development committee produced a standard and uniform system for evaluating PD in 1984 [30]. The average UPDRS score of 4.1 ± 1.2 reported.

The evaluation of PD patients in baseline and a 10-week follow-up condition was measured by the independent sample *t* test. The statistically significant chosen at *p* smaller than 0.05 data has been expressed by mean ± SD. In a 10-week follow-up evaluation, the stance duration was shown to be substantial, as was the slower speed gait in the baseline condition. The trunk fraction conditions were found significant in patients after rehabilitation training. The best response to rehabilitation treatment was seen when the trunk was rotated. Improvement > 5% was found optimal in trunk rotation.

Participants walked faster with 50° of chest flexure (TF2) in tranquil step (*p* of 0.01) and move-up (*p* of 0.05) than with regular upright posture (RE), according to a simple main effect analysis, though there were no within-step alterations when walking with regular erect trunk posture (*p* = 0.51), trunk flexure 1 (*p* of 0.05), or trunk flexure 2 (*p* of 0.01) (Figure 5). The standard deviation is indicated by the error bars. Here, *L* denotes for unperturbed level step; *U* − 1 represents preagitation step; *U* − 0 stands for step down; *U* + 1 represents step-up; RE illustrates the regular erect chest; TF1 stands for 30 chest dorsiflexion; TF2 denotes 50 chest dorsiflexion.

RETRACTED

Figure 6 shows the side-dependent time-distance characteristics. Statistically important differences are marked by asterisks (^∗^*p* less than 0.05; ^∗∗^*p* less than 0.01). We observed a critically higher number of group participants which recovered (all > 62%) than those who do not affect for each gait feature using a chi-square test. When GRF threshold characteristics are employed, mean accuracy improves by 52%. This considerable improvement in accuracy is crucial because, when no sigma-lognormal features were taken into consideration, it was possible to undertake an analysis utilising the interpatient separation scheme to discover who the poorly categorised steps belonged to. Regardless of gait posture, the step regular trunk flexure had significantly higher posture than the corresponding level steps, with a considerable rise in the 50 in trunk dorsiflexion 2 gait relative to the step “*L*.”

## 4. Discussion

Since chest-flexed locomotion is widespread (e.g., in the elderly people as well as people with spinal problems) has a negative impact on gait stability, it is important to understand how the trunk is involved in human locomotion. Based on stabilometric data, the study looked at postural stability in Parkinson disease patients when standing and walking in various settings. When compared to regular straight up walking, chest-flexed gaits across bumpy ground showed more stooping legs, defined by prolonged knee flex during stance. The TF1 and TF2 conditions were statistically significant among studied PD patients; these results were similar with Nag et al. (2011) study [32]. The use of this method with a more evident adaptation during trunk-flexed gaits is similar to how small birds handle significant terrain disturbances using their legs (i.e., a dodge-like formation) [28]. The duration of the gait cycle varies in a sophisticated way from one stride to the next, according on the computation of left and right foot stride signals. The “noisy” variations with stride signals of studied Parkinson diseased patients present from some fractal property (Table 5) [31]. Although it is far from the sole sign of PD, locomotor dysfunction is one of the most widespread [33].

RETRACTED

Although the stride monitor does not identify many more PD symptoms, including stiffness, difficulty swallowing, stooping posture, olfactory impairment, and upper-body rigidity and dyskinesias, there are few objective evaluations of these signs in the clinic. When the *p* values for *L* (unperturbed level step) and *U* + 1 (step-up) conditions were compared to the other conditions, the *p* values for *L* (unperturbed level step) and *U* + 1 (step-up) conditions showed a significant association with gait rhythm, implying that these two arithmetical parameters could be filtered as the leading features for the analysis of PD gait patterns. These findings demonstrate that in step *U* + 1, global leg kinematic changes and gait pattern were more step than posture dependent. The same gait database has been studied in a number of subsequent studies. Carletti et al. (2006) proposed a linear model to understand the stride interval time series in PD [34]. A linear regression model like this is suited for such single response problems [35]. They skipped the feature-correlation analysis, which is required before genuine recognition, because the statistical features of swing interval or stance interval were strongly related with those of stride interval.

According to our findings, patients with Parkinson's disease exhibit gait impairment, which is defined by decreased gait speed, reduced step length [36], decreased lower limb joint motion range, and considerably reduced trunk rotation in conjunction with an increased trunk rotation [37]. These findings suggest that rehabilitation should concentrate on the ground reaction force (GRF) metrics that are most sensitive to standardization, as well as substitute rehabilitative approaches for improving other parameters [38]. We also found the smallest clinically significant improvements in stereoisomerism and trunk rotation and dorsiflexion. Present research found that in people with Parkinson's disease, a reduction in stereoisomerism and geometrical irregularities ~25% and an improved performance in trunk spin and dorsiflexion ~10% above the duration of recuperation were medically useful and could lead to the standardization of these parameters, giving clinician thresholds to use when interpreting changes in gait parameters over time [39].

Clinicians are often given a single “snapshot” of a participant's neurological state, and PD therapy is commonly a trial-and-error technique that primarily relies on patient's subjective assessment to change the antidepressant dosage regime. Stride monitoring data over time might provide a more dependable and quick end-point. It is still challenging to create accurate and stable learning models from heterogeneous multisite data. Developing flexible algorithms and portable characteristics progressively over several locations to decrease intersite data variability might be a viable method.

RETRACTED

### 4.1. Limitation

Sample size and nonmulticentric are two major limitations of this study.

### 4.2. Future Scope

Clinicians are typically given a “snapshot” of a patient's motor state, and PD management is often a trial-and-error procedure that mostly depends on patient's subjective feedback to optimise the levodopa dose regime. Stride monitoring's long-term objective data may give a more fast and trustworthy end-point. Building accurate and stable learning models from heterogeneous multisite data is still a tough challenge. To reduce intersite data variability, developing adaptable classifiers and transferable features simultaneously across many sites might be a feasible method.

## 5. Conclusion

For patients with PD, mobility and gait difficulties are key concerns, and these clinical characteristics have an impact on their daily activities and social involvement. This study focussed on two major aspects, one is intervention, and second is gait assessment among patients suffering from Parkinson disorder. This study proves that there was some significant improvement observed in the gait parameters among patients with PD's which shows positive impact of the intervention. Also, here, we would like to suggest that such a sensor-based gait assessment may be considered part of an assessment battery and followed by auxiliary rehabilitative approaches especially for those who are more prone to improvement after short-term (10 weeks) rehabilitation in PD patients. This increases the reliability as reduces chances of human error in assessing the individual, since semiquantitative rating scale methods used to assess the performance and characterize of PD patients. Future Parkinson's disease research should shift away from laboratory-based studies of straight-line walking and more towards gait analysis in the home and community, where more complicated locomotor activities are severely hampered.

## Figures and Tables

**Figure 1:** Patient's recruitment process.

**Figure 2:** Gait cycle of normal human.

**Figure 3:** Flow chart describes patients' recruitment steps.

**Figure 4:** Flow chart describes the data acquisition method.

**Figure 5:** Steps and posture distribution measured during force exertion.

**Figure 6:** Gait analysis comparison in T0-baseline and T1-10-week follow-up. (a) Regular erect trunk, (b) TF1 (trunk dorsiflexion ~30°), (c) TF2 (trunk dorsiflexion ~50°).

**Table 1:** Hoehn and Yahr scale [19].

Stage 0:	No indication of disease
Stage 1:	One-sided indications (only one side)
Stage 1.5:	Unilateral symptoms in neck and spine
Stage 2:	Bilateral sides symptoms, but no loss of balance
Stage 2.5:	Mild sensations on bilateral sides that subside following the “pull” test (doctor ask the person to maintain balance while he pulls the man from behind)
Stage 3:	Mild or moderate illness, physical independence, and balance impairment
Stage 4:	Physical independence, balance issues, and mild to moderate illness are all factors to consider
Stage 5:	Unless supported, using a wheelchair or being bedridden

RETRACTED

**Table 2:** Hoehn and Yahr scale [19].

Stage 0:	No indication of disease
Stage 1:	One-sided indications (only one side)
Stage 1.5:	Unilateral symptoms in neck and spine
Stage 2:	Bilateral sides symptoms, but no loss of balance
Stage 2.5:	Mild sensations on bilateral sides that subside following the “pull” test (doctor ask the person to maintain balance while he pulls the man from behind)
Stage 3:	Mild or moderate illness, physical independence, and balance impairment
Stage 4:	Physical independence, balance issues, and mild to moderate illness are all factors to consider
Stage 5:	Unless supported, using a wheelchair or being bedridden

**Table 3:** Dataset for PD subjects with pull out characteristics.

Motion for right side feet	Motion for left side feet	Age	Height	Weight	Recorded time (second)	Speed of walking	BMI (kg/m^2^)
Gait time for motion vector (ms) -0.8753-0.4772	Gait time for motion vector (ms) -0.9761-0.5243	65-80 (years)	1.68-2.21 (meters)	45-101 (kg)	10 sec	0.6-1.75 (m/sec)	15.4-25.6

**Table 4:** Motor status discernment in Parkinson's disease patients.

Outcome	No. of patients	Beta	95% CI	*p* value	*R* ^2^
Age (65 ± 2.5)	25	0.042	2.8-4.5	0.05	-0.33
Hoehn and Yahr scale	25	0.006	0.82-0.12	0.527	0.37
Unified PD rating scale (UPDRS)	25.0	0.003	2.2-5.6	0.001	-0.23
Regular erect trunk	25	0.113	0.7-0.9	0.943	0.21
TF1 (trunk dorsiflexion ~30°)	25	0.056	3.8-6.7	0.005	-0.49
TF2 (trunk dorsiflexion ~50°)	25	0.001	2.5-4.7	0.001	-0.53

**Table 5:** Assessment of PD patients in baseline and a 10-week investigation state.

Parameters	Baseline				10-week follow-up assessment			
	Mean ± SD	*t*	*p*	Cohen's *d*	Mean ± SD	*t*	*p*	Cohen's *d*
Speed (m/s)	0.78 ± 0.29	-0.125	0.851	0.686	0.88 ± 0.12	-0.871	0.651	0.032
Stance duration	61.5 ± 3.4	-0.402	0.817	0.754	63.6 ± 2.2	-0.329	0.01	0.012
Step size (m)	0.15 ± 0.01	-8.012	0.750	0.629	0.16 ± 0.14	-13.65	0.391	3.301
Regular erect trunk	3.3 ± 1.6	-2.651	-3.146	<0.01	3.4 ± 0.12	-11.78	<0.001	2.761
TF1 (trunk dorsiflexion ~30°)	3.2 ± 1.3	-0.065	-0.637	0.934	4.0 ± 2.5	-12.69	0.015	0.745
TF2 (trunk dorsiflexion ~50°)	3.3 ± 1.0	-3.134	0.010	2.018	3.8 ± 0.65	-14.83	0.025	0.672

RETRACTED

## Data Availability

The data used to support the findings of this study are available from the corresponding author upon request.
